This article has been retracted.

# Relationship Between Chronic Kidney Disease Staging and Vitamin D Deficiency: A Retrospective Study

**DOI:** 10.7759/cureus.21221

**Published:** 2022-01-13

**Authors:** Theodosios Kantas, Camilo Andrés Avendaño Capriles, Sabir Babor, Tenzin Tamdin, Hady Al-Rihani, Anusha Thalla, Ahmed Adel Abdelmawla, Fares Mohammed Saeed Muthanna, Sohaib Tousif

**Affiliations:** 1 Surgery, Elpis - General Hospital of Athens, Athens, GRC; 2 Foundations of Clinical Research (FCR) Program, Harvard Medical School, Boston, USA; 3 Medicine, Universidad del Norte, Barranquilla, COL; 4 Medical School, Poznan University of Medical Sciences, Poznan, POL; 5 Medical School, Central America Health Sciences University, Ladyville, BLZ; 6 Surgery, Rafik Hariri University Hospital, Beirut, LBN; 7 Medicine, Katuri Medical College, Guntur, IND; 8 Department of Medicine, Aim Shams University, Cairo, EGY; 9 Pharmacy, Walailak University, Nakhon Si Thammarat, THA; 10 Medical School, Ziauddin Medical University, Karachi, PAK

**Keywords:** biomarkers, deficiency, staging, vitamin d, chronic kidney disease

## Abstract

Introduction

Vitamin D deficiency is a rising health issue in patients with chronic kidney disease (CKD). It can lead to serious issues such as rickets, periodontitis, osteoporosis, weakness, muscle ache, and depression. This study was conducted to determine the vitamin D status of patients with CKD in Pakistan and evaluate the correlation between serum vitamin D and renal function progression.

Methodology

A retrospective study enrolled patients who visited Liaquat National Hospital, Karachi, Pakistan, from January 2015 to January 2021 with a primary diagnosis of CKD. Anthropometric, laboratory, and demographic data were collected from the hospital management information system (HMIS).

Results

A total of 513 patients with CKD were included in the study. More than 50% of the patients were from stage 3 to stage 5 of CKD while the rest were from stage 1 and stage 2. Significant differences are in relation to calcium, phosphate, and albumin across categories of severity of CKD. Calcium is lowest in stage 5 while phosphate is highest in stage 5. Vitamin D deficiency was found in all participants, but serum vitamin D concentration was lowest in stage 5, i.e., 8.14+6.00. The changing of vitamin D level was associated with the severity of CKD staging (p-value=0.003).

Conclusion

The current study has shown that vitamin D deficiency, calcium deficiency, and hyperphosphatemia are more common in patients with CKD, but their severity is more common in advanced stages of CKD.

## Introduction

Chronic kidney disease (CKD) is referred to as kidney damage and reduced renal function that can be categorized into five stages as per the Kidney Disease Outcomes Quality Initiative (KDOQI) guidelines [1]. Globally, the prevalence of CKD was estimated at 13.4% [2]. People with CKD are experiencing an enhanced risk of cardiovascular disease, kidney failure, and death despite interventions to manage the risk factors. CKD has been identified as one of the world's most critical health issues, increasing global morbidity and mortality, while depleting scarce health resources [3]. As a result, better knowledge of its mechanism and new management strategies based on non-traditional risk variables are critical [4]. CKD is a risk factor for deficiency of vitamin D. It is common in patients with CKD, especially those with kidney transplant recipients and end-stage renal disease [5]. Vitamin D deficiency is present in all stages of CKD, and its prevalence is enhanced as renal function reduces [6]. Despite adjusting for CKD stage and confounding factors, people with vitamin D levels less than 15 ng/mL had an increased risk of all-cause mortality [7].

Vitamin D deficiency is a rising health issue in patients with CKD [8]. It can lead to serious rickets, periodontitis, osteoporosis, weakness, muscle ache, and depression [9]. Several studies have identified an association between vitamin D deficiency and reduced decreased glomerular filtration rate (GFR) in patients with CKD [10]. Vitamin D's importance in CKD goes beyond its traditional calcium and phosphorous homeostasis effects, including potential impacts on extra-mineral metabolisms such as immune system control and kidney function. According to certain research, vitamin D insufficiency in hemodialysis patients has been linked to muscle mass and strength [11].

In Pakistan, not many studies have been conducted to determine the association between vitamin D deficiency and CKD staging. Therefore, the treatment of CKD patients is often suboptimal or not well-targeted. Along with the deficiency of vitamin D, deficiency of inactive vitamin (nutritional vitamin D) is expected. Therefore, treatment needs to include active and nutritional vitamin D. In the case of early CKD, nutritional vitamin D is preferred [8]. Studying the pathophysiological role of vitamin D and discussing its association with CKD progression under various genetic backgrounds is critical. Therefore, this study has been conducted to determine the vitamin D status of patients with CKD in Pakistan and evaluate the correlation between serum vitamin D and renal function progression.

## Materials and methods

This was a retrospective study that enrolled patients who visited Liaquat National Hospital, Karachi, Pakistan, from January 2015 to January 2021 with a primary diagnosis of CKD. CKD is defined as abnormalities structure or function of a kidney that has been present for more than three months and has health implications (not graded). Overall, 590 patients visited Liaquat National Hospital, Karachi, Pakistan, from January 2015 to January 2021 with a primary diagnosis of CKD. Fifty-one (51; 8.64%) did not fulfill the eligibility criteria and data of 26 (4.40%) patients were missing. In total, 513 patients with CKD were included in the study.

The diagnostic thresholds were kept at an estimated glomerular filtration rate (eGFR) of less than 60 mL/min per 1.73 m^2^ and an albumin-creatinine ratio (ACR) of 30 mg/g or higher [12]. CKD was categorized into five stages as per the KDOQI guidelines, utilizing the estimated eGFR thresholds within the CKD range or evidence of changes in renal structures. Different stages of CKD and their eGFR values included stage 1 (eGFR ≥ 90), stage 2 (60 ≤ eGFR < 90), stage 3 (30 ≤ eGFR < 60), stage 4 (15 ≤ eGFR < 30), and stage 5 (eGFR < 15) [13].

Patients were not included in the final analysis if they had acute kidney injury (any of the following criteria: a urine volume < 0.5 ml/kg/h for six hours, increase in serum creatinine by ≥ 0.3 mg/dl within 48 h of hospital admission, age of less than 18 years, and history of bone-marrow transplantation or organ donation). Patients whose important data were missing were also excluded in the final analysis. All the variables were extracted from the hospital management information system (HMIS).

Anthropometric, laboratory, and demographic data were collected from HMIS by the investigator. Body mass index (BMI) was calculated as body weight (kg)/squared height (m^2^). Laboratory data at baseline included white blood cells (WBCs), hemoglobin, platelets, calcium, phosphate, albumin, cardiac reactive protein (CRP), parathyroid hormones (PTH), serum vitamin D, and creatinine were obtained from HMIS. eGFR was calculated by the CKD Epidemiology Collaboration (CKD-EPI) equation [14] using data extracted from HMIS.

Statistical analysis

Analysis was done using STATA version 16.0 (College Station, TX: StataCorp LLC.). Continuous variables were presented as mean and standard deviation while categorical variables were presented as frequency and percentage. The difference in the baseline characteristics of patients in five stages was determined using one-way analysis of variance (ANOVA) for continuous variables and the chi-square test of independence for categorical variables. Median and interquartile ranges were presented for hemoglobin, platelets, calcium, phosphate, albumin, c-reactive protein (CRP), parathyroid hormone (PTH), and their comparison was done in different stages of CKD using the Kruskal-Wallis test. Mean values were presented for vitamin D levels, and their association was seen with independent variables, including age, BMI, CKD, and gender using Pearson's coefficient, one-way ANOVA, and independent t-test as appropriate. Variables significantly associated with vitamin D are used to assess the relationship between CKD staging and vitamin D using multivariable linear regression analysis for controlling confounding variables. The correlation between estimated glomerular filtration rate (eGFR) and vitamin D was assessed using Pearson's correlation. A p-value of less than 0.05 was considered significant.

## Results

In total, 513 patients with CKD were included in the study. Based on the eGFR values, participants were assigned into five different stages as per the classification criteria discussed in the methodology section. The characteristics of participants by CKD stages are shown in Table 1. More than 50% of the patients were from stage 3 to stage 5 of CKD while the rest were from stage 1 and stage 2. Patients in the advanced stage were older than patients in the lower stages (p-value=0.008). No statistically significant difference was found between gender and CKD stages (p-value=0.411). BMI was also not statistically significantly different across different stages of CKD (p-value=0.057). Hemoglobin and platelets follow a decreasing trend in relation to the increasing severity of CKD, and statistically significant differences were found across the categories of severity (p-value<0.05). Significant differences were found in calcium, phosphate, and albumin across categories of severity of CKD. Calcium is lowest in stage 5 while phosphate is highest in stage 5. A significant difference was also reported in PTH levels among CKD staging (p-value=0.001). A weak and significant correlation was found between eGFR and serum vitamin D (r=0.018, p-value=0.012).

**Table 1:** Demographic and clinical characteristics of CKD patients * Significant at p-value <0.05 ^ Median (interquartile range) CKD: chronic kidney disease; BMI: body mass index; WBC: white blood cells; CRP: c-reactive protein; parathyroid hormone level; SD: standard deviation

Variable	Stage 1	Stage 2	Stage 3	Stage 4	Stage 5	P-value
Age (Mean (SD))	52.57 (14.85)	49.80 (13.61)	55.21 (11.44)	51.60 (15.15)	55.26 (15.79)	0.008*
Gender n(%)						
Male	34 (53.97)	53 (58.24)	42 (45.16)	66 (56.90)	81 (54.00)	0.411
Female	29 (46.03)	38 (41.76)	51 (54.84)	50 (43.10)	69 (46.00)	
BMI n(%)						
Underweight	12 (19.05)	7 (7.69)	8 (8.60)	12 (10.34)	24 (16.00)	0.057
Normal	16 (25.40)	43 (47.25)	33 (35.48)	48 (41.38)	55 (36.67)	
Overweight	15 (23.81)	22 (24.18)	27 (29.03)	38 (32.76)	36 (24.00)	
Obese	20 (31.75)	19 (20.88)	25 (26.88)	18 (15.52)	35 (23.33)	
WBC (109/L)^	6.11 (5.12-7.50)	6.41 (5.62-7.74)	6.50 (5.37-7.80)	6.22 (5.43-7.68)	7.08 (5.53-8.26)	0.1385
Platelets (1000/L)^	245 (202-276)	221 (195-256)	204 (178-240)	216.5 (184-255)	223 (183-265)	0.005*
Hemoglobin (g/dl)^	13.80 (13.30-14.70)	14.30 (13.10-15.60)	13.80 (12.50-15.30)	12.35 (10.95-13.95)	11.05 (10.3-12.1)	0.001*
Creatinine (mg/dl)^	1.00 (0.70-1.30)	1.10 (0.80-1.50)	1.20 (0.95-1.60)	1.20 (1.00-1.50)	1.30 (0.90-1.70)	0.001*
CRP (mg/dl)^	0.04 (0.02-0.093)	0.05 (0.02-0.17)	0.06 (0.03-0.12)	0.07 (0.04-0.15)	0.05 (0.03-0.19)	0.516
Calcium (mg/dl)^	9.20 (8.80-9.80)	9.30 (8.80-9.50)	9.20 (8.70-9.60)	9.10 (8.60-9.60)	8.90 (8.40-9.40)	0.001*
Phosphate (mg/dl)^	4.05 (3.55-4.75)	4.10 (3.60-4.80)	4.10 (3.50-4.70)	4.45 (3.75-4.65)	4.9 (4.20-5.80)	0.001*
Albumin (g/L)^	4.00 (3.40-4.60)	4.10 (3.50-4.70)	3.90 (3.40-4.40)	4.45 (3.75-4.65)	4.90 (4.20-5.80)	0.001*
PTH (pg/ml)^	13.10 (7.20-23.60)	7.50 (59.00-11.40)	8.60 (5.60-13.20)	16.00 (8.70-26.1)	22.80 (14.60-31.40)	0.001*

Hypertension was the most common comorbidity found among patients in the current study, followed by diabetes. Hypertension and diabetes were present among 80.31% and 70.37% of patients, respectively. The frequency of hypertension and diabetes are significantly higher in advanced stages than in lower stages (p-value<0.05). The incidence of all other comorbidities is significantly low and no significant difference was found in different stages as shown in Table 2.

**Table 2:** Common comorbidities in CKD patients at different stages *Significant at p-value<0.05 Presented as n (%) CKD: chronic kidney disease

Comorbidity	Stage 1	Stage 2	Stage 3	Stage 4	Stage 5	P-value
Diabetes mellitus	38 (60.31)	54 (59.34)	65 (69.89)	86 (74.13)	118 (78.67)	0.001*
Hypertension	43 (68.25)	70 (76.92)	73 (78.49)	95 (81.89)	131 (87.33)	0.001*
Ischemic heart disease	4 (6.78)	9 (10.34)	8 (8.79)	10 (9.09)	11 (7.75)	0.911
Liver disease	7 (11.11)	10 (10.99)	9 (9.67)	12 (10.34)	11 (7.33)	0.155
Respiratory disease	4 (6.35)	6 (6.59)	9 (9.67)	10 (8.62)	8 (5.33)	0.266
Gastrointenstinal disease	8 (12.69)	13 (14.28)	13 (13.97)	18 (15.51)	22 (14.67)	0.561
Others	6 (9.52)	10 (10.99)	8 (8.60)	8 (6.89)	12 (8.00)	0.641

Table 3 lists details of the univariate analysis and multiple linear regression between serum levels of vitamin D and staging of CKD and shows the serum concentration of vitamin D in stages of CKD. Vitamin D deficiency was found in all of the participants, but serum vitamin D concentration was lowest in stage 5, i.e., 8.14+/-6.00. The changing of vitamin D level was associated with the severity of CKD staging (p-value=0.003). Other factors significantly associated with serum vitamin D concentration among CKD patients included age (p-value=0.037), gender (p-value=0.001), and BMI (p-value=0.006). A post-hoc Tukey's test shows that vitamin D level is significantly different in stage 5 as compared to stage 1, stage 2, stage 3, and stage 4. The post-hoc Tukey's test was also applied to see the differences of vitamin D in BMI groups. A significant difference is reported in vitamin D levels between normal and obese patients.

**Table 3:** Relationship between vitamin D level and independent variables * Significant at p-value<0.05 ^ Correlation coefficient (r) A post-hoc Tukey's test was applied to compare the mean of each category in CKD staging and BMI. Means not sharing subscripts differ significantly at p-value<0.05 as indicated by the post-hoc Tukey's test. SD: standard deviation; CKD: chronic kidney disease

Variable	Vitamin D (ng/ml) Mean (SD)	P-value
CKD staging		
Stage 1	16.00 (8.42)a	0.003*
Stage 2	15.65 (5.58)a	
Stage 3	11.40 (6.14)a	
Stage 4	11.76 (9.87)a	
Stage 5	8.14 (6.00)b	
Age of participant^	-0.091	0.037*
Gender		
Male	12.51 (6.87)	0.006*
Female	9.37 (8.94)	
BMI		
Underweight	9.93 (5.18)b,c	0.001*
Normal	12.69 (7.82)b	
Overweight	10.58 (6.05)b,c	
Obese	9.54 (10.58)c	

Variables significant in univariate analysis were used to generate the final model using multivariable linear regression analysis. Table 4 shows that a vitamin D deficiency is significantly greater in patients with advanced CKD staging than in lower staging after adjusting all other confounding variables.

**Table 4:** Multivariable linear regression analysis between serum vitamin D level and CKD staging CI: confidence interval; CKD: chronic kidney disease

Variable	B-coefficient (95% CI)	p-value
CKD staging		
Stage 1	3.75 (0.83,6.68)	0.012
Stage 2	3.28 (0.48,6.07)	0.022
Stage 3	2.50 (-0.56,5.58)	0.109
Stage 4	3.21 (0.17,6.25)	0.038
Stage 5	Reference	
Age of participant^	-0.008 (-0.014,-0.003)	0.001

## Discussion

CKD has become a major public health issue worldwide, particularly in developing countries. In Pakistan, the prevalence of CKD among adults was 21.2% [15]. Our study findings demonstrated that mean age is greater in patients with a more advanced stage of CKD. The study conducted in China in 2012 found that the average age of patients with CKD at stages 3 to 5 is higher than the average age of patients with CKD at stages 1 to 2 [3].

Diabetes and hypertension are common comorbidities among CKD patients in the current study. CKD is a consequence of uncontrolled hypertension and a prevalent cause of hypertension. The hypertension prevalence in CKD patients could rise from 68% to 87%, along with declining eGFR in advanced stages. The study conducted by Wang et al. also reported similar findings in which the prevalence of hypertension in CKD stage 1 patients was 67% compared to the 92% in CKD stage 5 patients [16]. Besides this, the prevalence of diabetes mellitus is also higher in patients with advanced CKD staging, and similar findings were also reported in the study conducted by Wang et al. [16].

In CKD, vitamin D deficiency is frequent, and it is linked to the increasing increase in PTH that occurs as renal function declines. It can also increase cardiovascular risk, mineral bone disease, and hyperparathyroidism [17]. Our study has found that deficiency of vitamin D was present among all patients enrolled in the current study. Still, the deficiency is more severe in advanced-stage patients than in lower stages. Deficiency of vitamin D is as high as 80 percent in patients with CKD, which has been linked to albuminuria, quicker kidney disease progression, and higher all-cause mortality [18].

A weak positive correlation between eGFR and vitamin D was reported in the current study, similar to the study conducted by Wang et al. [16]. It indicates that the concentration of circulating vitamin D is lower in patients at advanced stages of CKD. Deficiency of vitamin D can be related to reduced food intake, insufficient vitamin D3 from 7-DHC [19], and inadequate exposure to sunlight. Because of the limitations of the study design in this research, it was difficult to assess the role of the above-mentioned factors in vitamin D deficiency. As deficiency of vitamin D can lead to poor outcomes among patients with CKD, such as the increased risk of mortality [20], physicians need to emphasize the importance of the management of vitamin D concentration among patients with CKD.

In this study, we have also compared the calcium, phosphate, and albumin levels in five stages of CKD. The findings showed a deficiency of calcium in advanced stages of CKD while phosphorus is in the normal range in stage 1 to stage 4 of CKD. In contrast, stage 5 has a significantly higher serum phosphorus level. Considering the impact of CKD staging on calcium and phosphate, correction of hyperphosphatemia and hypocalcemia should be addressed as a preliminary step. Calcitriol can be used to treat secondary hyperparathyroidism caused by CKD [21]. PTH, as well as serum phosphate and calcium, should be checked on a regular basis. KDIGO 2017 guidelines mention that the serum calcium, parathyroid hormone (PTH), and phosphate levels should be monitored in every CKD stage, and treatment needs to be based on serial assessments of PTH, calcium, and phosphate levels, considered together [13]. It is worth noting that the optimal PTH range for dialysis patients is two to nine times the upper normal limit, whereas the best range for non-dialysis patients is unknown. If there is a downward or upward trend in values, treatment should be adjusted to reverse the negative tendencies [22].

The current study has certain limitations. First, data related to vitamin medications, vitamin supplements, enteral feeds, and dietary intake related to mineral and bone metabolism of patients were missing, making it difficult to analyze etiologic hypotheses. Second, it was a retrospective study; therefore, we were not able to analyze several other factors as well. Third, it used the data of only one tertiary care hospital. In the future, more prospective multicenter studies need to be conducted with a larger sample size, including inpatients and outpatients, to get more generalizable findings and reduce confounding factors and possible biases. Finally, we were not able to determine the causes of CKD among the patients in the current study.

## Conclusions

The current study has shown that vitamin D deficiency, calcium deficiency, and hyperphosphatemia are more common in patients with CKD. Still, their severity is more common in advanced stages of CKD. Health care professionals should educate and counsel CKD patients regarding nutritional sources of vitamin D and its monitoring. Primary care physicians are being urged to join nephrologists, endocrinologists, nutritionists, other specialists, and public health agencies in disseminating and implementing updated guidelines and recommendations to combat the growing epidemic of vitamin D deficiency, especially among the highly vulnerable CKD population.
